RETRACTED

# On the Feasibility of Integrating the Concept of Contemporary Green Environment Development in Creating Screen Prints by Digital Means

**DOI:** 10.1155/2022/3938915

**Published:** 2022-10-04

**Authors:** Lei Xue

**Affiliations:** School of Fine Arts, Zhejiang Normal University, Jinhua, Zhejiang 321004, China

## Abstract

In the 21st century with the popularization of digital technology, as a printmaking born out of industrial printing, it has undergone a revolutionary evolution. Silkscreen printmaking is a type of print with high technology content, strong dependence on media, and no traditional load. Thirty years ago, as soon as silkscreen prints settled in China, they began artistic exploration and experimentation with a brand-new attitude. Several generations of screen print workers have achieved it, expanded it, and made it independent in the fusion of modern language methods and oriental cultural spirit, and in the exploration of screen vocabulary, characteristics and character, it has an independent status and ranks among the international elite qualifications. This paper analyzes the root problems of high-tech printmaking tools, materials, technical principles, and causes of aesthetics. Starting from the background of the concept of green development, it expounds its related concepts, analyzes the theoretical origin of green development, and clearly recognizes the high-tech. The limitation of printmaking in the development space—that is, the expression language of digital plate making, is relatively correct in theory, so as to carry out step-by-step exploration and practice.

## 1. Introduction

In the printmaking family, silkscreen prints are a type of painting with high technology content and strong dependence on media [1]. The expression form is relatively free, with a strong sense of the times and design [2]. Like the generation and development of other types of prints, the development of silkscreen prints has also gone through the process from practical printing to artistic creation [3]. The forms of images are rich, and there are various image processing methods such as hand-painted, produced, copied, and digital computer synthesis. Painters choose and arrange pictures according to their own creative ideas, so that the images can better express the personality and thinking of the works and more closely express the theme of creation. The advantages of screen prints are reflected in the processing and control of color, which determines the unique limitation of the expression language of prints [4].

In this sense, the color of screen printing is not the color overlapping and mixing in the general sense, but the combination and composition of the overall pattern color [5]. First of all, under the guidance of creative ideas, the color and structure of the graphics can be judged after referring to the materials, clarifying the expression method, and determining the modeling mode of the graphics [6]. The color here refers to two levels: one is the overall effect of color juxtaposition and superposition of images; the second is the color contrast, which is divided into cold and warm, light and dark, purity and grayscale [7]. The structural relationship refers to the cooperation relationship between the picture and the image and refers to the organic combination relationship of the points, lines, planes, bodies, and other elements that constitute the image, that is, the overall structure of the interrelationship between the picture and the image [8]. The visual effect brought by the sense of artistic form is the embodiment of the artist's ideas [9]. With the development of the times, high-tech digital technology has greatly facilitated the production of screen prints and also enriched the expression language of screen prints [10]. With its strong industrial and design sense, screen prints naturally integrate digital technology. Absorb it as its own expressive technique [11].

RETRACTED

A variety of application software can be selected in the digital production process, such as image processing application software: Adobe Photoshop, paint, Corel photo paint, etc.; and famous graphics processing software: Adobe Illustrator, CorelDRAW, etc. In addition, 3D modeling and rendering software such as 3DMAX can also be used [12]. Take advantage of with the support of many application software, the powerful functions of computers can be described as all-encompassing, but the process of digitization belongs to the process of logical thinking after all. What it lacks is the abstract thinking ability of human beings. Fortunately, computers are controlled by us. It is our tool for artistic creation—just a tool, a super tool driven by human creative thinking, which is the beauty of digital art.

With the rapid development of the economy, excessive energy consumption has caused a shortage of various resources, resulting in “ecological problems” [13]. This problem manifests itself primarily through the buildings and environments in which we live [14]. In order to save energy, relevant scholars put forward the concept of green building, that is, buildings should reduce environmental degradation through technology. It is a new architectural model of symbiosis, coexistence, and sustainable development of people, environment, and architecture and has the characteristics of sustainable development. In order to build an ecological civilization, the party's “Ten Great Goals” put the building of an environment-friendly, energy-saving, and emission-reduction society at a prominent position in the modernization and industrialization development strategy. Promoting green urbanization and building an innovative city is an important measure for my country to implement the scientific concept of development and sustainable development. Building energy consumption, industrial energy consumption, and transportation energy consumption are the main components of total social energy consumption. Therefore, in order to implement the spirit of the national energy conservation and emission-reduction policy, it is imperative to develop green buildings [15]. The so-called green building refers to saving resources (land saving, energy saving, water saving, and material saving) to the greatest extent, protecting the environment and reducing pollution during the whole life cycle of the building, and providing people with healthy, applicable, and efficient use of space architectural forms that coexist in harmony with nature. Green building emphasizes “four sections and two environmental protection” [16]. The so-called “two environmental protection” includes the following two meanings: the first is to protect the external ecological environment to minimize the disturbance to nature; the second is to protect the indoor environment and improve the health of the occupants [17].

RETRACTED

Designing a sustainable and low-energy living environment is the development trend of today's interior design [18]. The realization of sustainable development is usually achieved through the following two ways: (1) improving the energy efficiency by improving the infrastructure construction; and (2) changing the behavior of the occupants through interior design [19]. To achieve this goal of green interior design, interior designers need to have a new way of thinking to conduct research and practice for our next generation of interior designers [20].

## 2. Current Situation of Silkscreen Printmaking

### 2.1. The Ecological Environment of Contemporary Chinese Silkscreen Printmaking

The creation and spread of blackboard writing has a long and glorious history in the history of Chinese art. The rise and fall of Chinese fine arts have a direct and inevitable relationship with the social and economic development of various countries and local governments in the world. With the development of industrial science and technology and the gradual improvement of the country's comprehensive national strength, silk screen printing art was born on the art stage of China with the bell of China's reform and opening up. Good social conditions and open-minded cultural attitude have created an infinite and broad living space for its vigorous development. Chinese screen printing is a kind of printing with high technical content, strong dependence on media, no cultural precipitation, and no cultural load. When screen printing was just settled in China's domestic universities, it was carrying out cultural innovation and development in a brand-new state. Therefore, although China's silk screen printing has a history of more than 30 years, they can be said to be colorful from their inception to the present.

RETRACTED

With the struggle of a generation of silk screen printing workers, China's confidence, courage, and strength have been developed and developed in the integration of modern language technology and oriental culture and art, making it independent. In the field of screen vocabulary and language research, China has its own advantages and international qualifications. Digital technology and other emerging media have opened a new era of their development. With the development of science and technology, the improvement of production equipment and conditions, and the entry of a large number of foreign media, screen printing has changed its environment, changed its communication methods, and improved its production level, thus promoting its own modernization development.

However, after all, the history of silk screen prints is still short, and the research on its ontology language characteristics, advantages, and creation laws is not enough. In addition, in the traditional Chinese art education system, there are still some problems in the teaching content and social needs. Barriers to teaching or printing still exist; there is a lack of academic research on how to take the pure print technology as the social needs of their own growth after graduation; the school has no conditions for professional print studio; based on the social characteristics of print works, college students who are separated from the school working environment cannot create print; because the students' personal creative value is high, they do not have a school working environment, or they do not have enough understanding of print works, so other print artists rarely consider creating prints; the basic industries such as galleries have biased understanding of printmaking products, while the industry's understanding of printmaking technology is imperfect, and the loss of production talents is also caused by social conditions; the distinction between original print works, copy print works, and decorative paintings is also vague; under the guidance of the artist studio system, there is a lack of multitype and multilevel print creation activities in international professional large-scale exhibitions; and the lack of printmaking materials. A series of social problems have formed the main obstacles to the development of printmaking art and also caused the slow development of contemporary Chinese printmaking art while flourishing in social culture and economy as shown in Figure 1.

RETRACTED

### 2.2. The Technical Characteristics and Language Expression of Digital Technology Prints

The creation of digital plate making faces two extremes. First, digital technology plate making has the basis of delicate expressiveness, which makes it extremely capable of reproducing figurative themes. However, many authors seem to treat high-tech prints with traditional printmaking concepts. For example, in silkscreen prints, they confuse the concept of imprint and print mark and think that as long as the traces formed on the paper by the paint leaked through the silkscreen are silkscreen prints, they have embarked on the idea of reproducing the image of the object, but this way going down, whether it is the color gradation version or the CMYK film version, it is limited to the concept of replicating objects, and in the era of digital products, any mobile phone is equipped with a camera of 1 million or 10 million pixels. The advanced computer makes it easy for people to be satisfied with the aesthetics that exist in the objective image. Therefore, the visual works that over-reduce the image are unbearable in terms of efficiency and price.

Secondly, the delicate expressive power of digital technology plate making makes it omnipotent, and omnipotence also means at the same time nowhere. Therefore, the youngest silk screen prints seem to inevitably go to another creative extreme on the road of exploration—pure. The combination of principled visual mode, abstract image, and new sense of form is refreshing, but today, 70 years after the death of Kandinsky and Mondrian, is this creation or repetition? Screen printers are a lonely group, and there is a certain distance between screen prints and contemporary cultural forms, which makes screen prints seem to be talking to themselves. As a result, the aesthetic value of silkscreen prints returns to its unique language limitations without any suspense: namely, texture expression, and the special superposition method that exists in conjunction with texture expression, as shown in Table 1.

### 2.3. Concept of Green Development

China's green development concept is put forward on the basis of conforming to the inevitable law of human development. It is a comprehensive summary of global development and determines the new goals of China's ecological and social development, as shown in Figure 2. The idea of green civilization is mainly to encourage human beings to establish green values, green culture, and survival mode. Its ultimate goal is to make human beings achieve natural harmony. Our values are the foundation of green economy. The concept of green development is based on respecting and understanding nature and its laws. The main purpose is to serve people's future development. It is no longer at the cost of damaging the natural environment, but for common development—mutual harmony. Under the environmental requirements of continuous adaptation and survival and development, people will develop resources according to the social reality and will strive to maintain resources, so that human beings can achieve the broadest development in society both materially and spiritually. The concept of green development advocates harmonious social values in all aspects, which is an important theoretical cornerstone and spiritual power to promote human green development.

RETRACTED

In May 2017, during the forty-first collective study of the Political Bureau of the CPC Central Committee, Xi Jinping proposed that to provide people with an excellent environment for people to produce and live in, it is necessary to promote green development and life ways. The concept of green development requires a change in the way of development and must give up the form of development that is harmful or even damaging to the environment. It is wrong to not only see temporary benefits and go for a short-term economic rise to infringe on the ecological environment. (1) Adhere to the people as the main body, the concept of green development is to achieve people's ecological happiness as the goal and to improve people's living standards and quality through green development. “The environment is the livelihood of the people, the green mountains are beautiful, and the blue sky is happiness.” (2) The purpose is to allow the people to obtain ecological happiness and achieve social benefits.

The final result of green development should benefit the general public. To effectively promote green economic development, we should start with the vital interests of the people, create a good living environment for the people, ensure the basic living requirements, and improve the people's living taste and quality of life. Make it the foundation of a good life for people. The concept of green development adheres to the fundamental aspirations of the people, what kind of living environment the people pursue, and what kind of ecological guarantee the concept of green development should provide. Feature the characteristics that conform to the human's expectations for a better life and realizing their ecological happiness is the value purpose of the green development concept. It is necessary to always take people's requirements as the goal and way of development. The goal is to enable people to live an ideal life and satisfy people's pursuit and yearning for a happy life. This is also the value characteristic of green development.

RETRACTED

## 3. The Application of Digital Technology in the Creation of Silkscreen Prints

### 3.1. Sketching Stage

When we have an idea, we need to visualize the thinking image. Usually, we describe it on paper, which is a “sketch”. We can also introduce digital technology, use digital cameras, scanners, and other digital devices to digitize hand drawn sketches and other digital materials, and then use powerful computer adjustment and editing functions for digital reconstruction, or draw directly with a mouse or light pen.

Compared with traditional creation methods, digital creation has many conveniences: (1) the traditional tools such as paper, ink, pen, and color are omitted, and everything is on the screen. The powerful brushes and palette tools provided by the drawing software can be used as it is more convenient. (2) Tone adjustment, color conversion, and adjustment tools such as copying, stretching, moving, rotating, and cutting provided by the drawing software can modify the drawing at will, which is faster. (3) The drawing software has rich special effects. The filter tool allows us to make more attempts and display the results directly on the screen, what we think is what we see. (4) It can make full use of the massive material resources provided by the image CD and the Internet, which greatly expands the creative space. (5) We can save any display result as an electronic drawing file, which is convenient for future reference, comparison, and modification and can also be printed out on paper to turn it into an actual, traditional “sketching.” (6) For printmakers, the advantages of digital technology do not stop there. The specific process is shown in Figure 3. There are many functions of the drawing software that are specially designed for the printing industry. The final result of printmaking is also realized through printing. The settings of layers, channels, and spot colors are used for the printing of prints and have special meaning.

### 3.2. Creation Stage

The digital creation stage of silkscreen prints is to use digital means to deeply describe the selected drafts, determine the number of sets, printing sequences and printing processes (paper, ink, plate making methods, mesh specifications, etc.), and print them in accordance with the whole process of color separation processing on the image file, and finally, outputting the required positive image transparencies. Most of the work in the stage of printmaking is to make printing plates for printing, and different types of plates use different materials, tools, and production methods. Screen prints use the silk mesh cloth taut on the frame as the printing plate, use various plate making methods to consciously block the partial mesh holes, and use the pressure of the squeegee to make the ink leak through the unblocked mesh holes to the screen imprints form on the paper.

RETRACTED

Among the many plate-making methods of screen printing, the photosensitive plate-making method is currently the most widely used. After that, the screen plate required for printing is obtained, and the black positive image part on the transparent film that blocks the light is the final imprint. Therefore, the creation of silk screen printing is largely the production of the positive image transparent film used for plate making. The production of positive image transparencies can be done digitally.

### 3.3. Printing Stage

The printing of silk screen prints is mostly manual, and the printing process itself is also a process of continuous creation, as shown in Table 2. Because automatic equipment is generally not used, the use of digital technology is less, but we can still use the predictive function of the computer to provide some useful help for the printing of prints. In the printing process of screen prints, due to uncertain factors such as the characteristics of paper, the characteristics of ink, the addition of auxiliary materials, the conditions of the printing environment, and the size of manual pressure, the final result will be slightly deviated, sometimes even have some unexpected special effects that will appear. Use the computer to adjust the results in real time according to the actual situation and make real-time predictions for the next printing plate, which is of great help to improve the quality of the work.

Using the photosensitive method for plate making, first convert the original into an electronic manuscript. Color originals should be screened by C, M, Y, and K. Generally, refer to Table 3 for the screening angle, which can effectively eliminate moiré. Then output the negatives, respectively, check the discrepancies with the originals, and use them as printing plates after trimming.

The practical significance of computer application is to make digital technology produce artistry, so as to serve the creation of silk screen art, so as to achieve the practical value of digital technology in silk screen printing. According to the first draft, plate making, printing in order on this basis, and finally make appropriate adjustments. In the design of the entire operation process, try to be reasonable and scientific. Therefore, the first draft of creation should be carefully prepared, the space division and printing sequence should be organized, and the artist's creative thinking and writing motivation should be fully expressed as far as possible; in the printing process, the gap should be adjusted in time to master the best accidental results; in the adjustment stage, the integrity of the image should be taken into account as much as possible to highlight the core of the image and make the painting rich and harmonious.

RETRACTED

Although silk screen printing has a development history of nearly 20 years in China, it promotes China's own modernization with brand-new concepts, rapid contact with new things, emphasis on physical discovery, three context transformation, pattern innovation, and skill improvement. However, after all, the development history of Chinese silk screen prints is still very short. In addition, the in-depth study on the characteristics and advantages of its ontological language and its creation laws is not enough. This new type of print has always been in a plain state. How to deal with the relationship between thought transmission and artistic feeling, knowledge and creation, printing effect and reproduction tendency, how to give full play to its modeling and design function, and how to deal with the relationship with general art and fine arts, put it in front of the screen printing industry.

## 4. Reflections on Screen Prints under the Trend of Green Development Concepts

The natural environment is the basis for people's survival and development, and cannot be replaced by any item. The green environment in a broad sense refers to the sum of environmental elements composed of material and nonmaterial factors. Among them, the material factors refer to such naturally existing factors as the atmosphere, soil, water, animals, and plants, while the nonmaterial factors refer to some ideologies, mainly the concepts and laws of the environment. In a narrow sense, green environment refers to factors that can meet people's requirements for survival, and can be in harmony with ecology and the environment, such as clean land, clean air, and water resources. The combination of these factors is a green environment, such as Figure 4.

The concept of green environmental development emphasizes the protection of the natural environment and the earth's creatures and advocates that by using natural resources effectively and to a certain extent; we can further improve the environment for people to live in nature and promote human activities to be compatible with nature. The environment in the environment checks and balances each other to achieve a stable state, so as to achieve the effective common development of any natural whole. Nowadays, the problem of ecological environment is becoming more and more serious, and it is more urgent to strengthen the ecological awareness of the people and establish a correct concept of green environmental development.

RETRACTED

### 4.1. Will the Development of Digital Prints Replace Silkscreen Prints?

Digital printmaking is developed in a specific scientific and social environment and can also be called digital printmaking and computer printmaking. The language of artistic expression is different from the imprint language of screen prints. The artistic creation of digital prints mainly relies on computers and printers, and the ontology language of screen prints is the artistic expression based on prints, which is also different from the basic language of digital prints feature. Although, some new features produced by the application of digital technology to the creation of silkscreen prints are similar to the basic characteristics of digital printmaking, the unique language charm of silkscreen printmaking is missing from the context of digital printmaking itself. The soul of the screen print. The artist Xu Bing believes: “Printmaking is an indirect painting, it is through the artist's intention to prescribe the treatment of the medium, and through the indirect process of printing, the medium is transformed into traces and presented as a picture.”

The performance of the screen print is presented through the imprints of various techniques. It can be said that without the existence of the imprint, the charm of the screen print will cease to exist. The expressiveness of digital prints is completely presented through high-tech digital language, and the level of pixel quality naturally becomes the unique digital language charm. In terms of artistic charm, digital prints and screen prints do not conflict. The rapid development of science and technology and the continuous innovation of art make it easy for some artists to lose their original intention of creation, and it is easy to go into misunderstandings in terms of techniques. Too much pursuit of schemas and too much catering to the society will lose the value of art. Digital prints and screen prints have their own characteristics. Digital technology plus screen prints and digital prints are not equal. Whether you choose screen print creation or digital print creation, they should be different from the art of the work. Expressive and unique printmaking charm make full use of their respective language characteristics to create printmaking works full of era significance.

RETRACTED

### 4.2. Can Silkscreen Prints Usher in New Business Opportunities under the Integration of Digital Technology and Green Development Concepts

Green environment is the soul of green development. It revolves around green development from beginning to end and is an aspect of green development that cannot be ignored. In the process of green development, green environment exists as a guiding function, as shown in Figure 5. Green environment is the environmental premise of green development. Without it, green development cannot be mentioned. Green environment is such a harmonious relationship that reflects any nature, which contains a variety of ways and concepts etc. People live in the environment and want to get good development and living space, then they must rely on the green environment as if the ecological environment is damaged, the resources and environment will also become an obstacle to green development, which hinders the overall construction of a well-off society and basic modernization.

Green development is a sustainable development. Its central meaning is to put the environment in the most prominent part and integrate it into all aspects of society according to its requirements, so as to gradually realize the common progress of both the environment, ecology, and society. This is also green. The importance of the environment in development. If the green environment is lost, the green development will be lost, let alone the continuous development of the society. With the development of economic society, aesthetic economy, and commodity economy, silk screen prints were originally a category of art, but today they have quietly infiltrated into commerce and created more value than themselves. In today's era of the prevalence of e-commerce, the emergence of various self-media has increased the activity of silk screen prints in the business world. In today's developed Internet, how to integrate the combination of art and business and effectively give full play to them, the real value of each other to achieve the maximum benefit of the combination of the two is a question worthy of our consideration. Today, in this fast-developing era, silkscreen prints are widely used in our lives. The reason why printmaking is widely used in modern life is that printmaking has characteristics that other types of painting do not have, such as the reproduction characteristics of printmaking. As an art painting, it can have many original works. A painting is the original version, such as oil painting, Chinese painting, and watercolor, which do not have such advantages.

## 5. Conclusion

Green technology plays a pivotal role in development. It must comply with the requirements of green development, promote development in an all-round way, and at the same time, keep pace with the times and possess advanced green technology. With the support of green technology, the green economy can better provide impetus for green development and promote the process of green development. Whether it is the social structure form or the artistic culture form, its essence is an organic natural pattern. Each form of artistic expression needs to grow reasonably and rapidly in a suitable natural environment, and in a natural environment that does not have reasonable growth requirements, people must make corresponding adjustments and adaptations to their own development. From the spontaneous individual development in the past to the development of the overall growth in the future, as well as the development of modern silk screen printing, such collision and correction will inevitably occur, so as to meet the ever-changing needs of the development of information media technology.

RETRACTED

## Figures and Tables

**Figure 1:** Research trend of silkscreen prints.

**Figure 2:** Scatter plot of environmental decentralization and green development.

**Figure 3:** Flow chart of digital technology for making silkscreen prints.

**Figure 4:** Composition of the natural environment.

**Figure 5:** The basic process and market trend of silk screen printing.

**Table 1:** Comparison of technical parameters of various prints.

Category	Requirements of the environment	Environmental requirements	The technical requirements	The cost	The efficiency	Artistic reproduction effect	Repeatability
Silk screen print	The print is made into a screen in which the blank part is blocked, and the text part is ink-permeable	The production technology and conditions are higher	Have certain printing background, can operate all kinds of equipment skillfully	Low	High	Rich color and strong display	High

Black and white woodcut	The blank part will be removed on the board, leaving the raised text part	Moisture proof	Pay attention to three tastes (knife taste, wood taste, and seal taste)	The cost of general	Middle	Black and white composition	Middle

Woodcut tinted	Multicolor engraving and printing	Less demanding	Weaken knife technique and pay attention to color harmony	The cost of general	Middle	Color coordination, strengthen gray bar application	Low

Watermark wood	Using cellophane paper to transfer the original manuscript to a wooden board in the process of engraving	High requirements for air humidity	The layout cannot water, paper to maintain a certain humidity	The cost of general	Middle	Elegant, solemn, strong tone	Middle

Copperplate engravings	Etching or engraving of copper or zinc plates	Special tools and facilities are needed	Paper required 180-250 grams, pay attention to ink viscosity	The cost is high and the process is tedious	Low	Soft, delicate, strong visual impact	High

Lithographic prints	The original manuscript was painted on a stone slab and corroded to form a stone plate	A dedicated lithographic studio is required	Corrosion control, ink balance in the printing process	The cost is high and the process is tedious	Low	Artistic reproduction effect	High

RETRACTED

**Table 2:** The plate-making process of the three major plate-making methods.

Category		Plate-making process
Manual imaging plate making	Hand-painted legal version	In the clean screen, the use of Arabic gum is directly painted, dry after the full plate coated with shellac, and then the printing plate immersed in the temperature of 50-60°C in water, after the Arabic gum melted, the graphic part is exposed, blank part of the mesh is shellac-blocked
	Plate making by cutting	On the paper or transparent plastic evenly coated shellac thickness in 3-5 mm, dry in the film to depict the manuscript, and then through overheating, transfer the manuscript to the net cloth
	Sealing method version	Draw the drawing ray wants to print on the stretched mesh, andthen use the pen to fill in the blanks

Photosensitive imaging plate making	Engraving film and plate making	A hollow-out mold is carved on the film, and then the mold is pasted on the screen to form a printing plate
	Direct plate-making method	In the stretched net cloth coated with photographic glue, and then paste on the film, exposure, development, drying, and other processes, the final formation of a printing plate
	Indirect plate making method	Using positive negative for exposure and development, and then transferred to the mesh, plug hole, sheet base stripping, and forming of a printing plate

Digital imaging plate making	Straight plate making	In the dry mesh on the photosensitive film, and then coated with photosensitive adhesive, film base stripping, combined with positive negative exposure and image production plate

**Table 3:** Screening angle reference table.

Type	C (○)	M (○)	Y (○)	K (○)
Monochromatic	45	45	45	45
Double color		Dark 45, light 75		
Three color	45	75	15	
Four color	75	15	0	45

## Data Availability

The labeled data set used to support the findings of this study is available from the corresponding author upon request.
